The article "Hepatolithiasis associated with intrahepatic heterotopic pancreas: a case report and literature review" was published in 2015. Journal: Diagn Pathol.

# Hepatolithiasis associated with intrahepatic heterotopic pancreas: a case report and literature review

**DOI:** 10.1186/s13000-015-0319-8

**Published:** 2015-06-23

**Authors:** Zhi-Yong Yu, Zhong-Quan Sun, Min Zhang, Bei Wang, Wen Lu, Shu-Sen Zheng

**Affiliations:** Division of Hepatobiliary and Pancreatic Surgery, Department of Surgery, First Affiliated Hospital, Zhejing University School of Medicine, Hangzhou, 310003 Zhejing Province China; Department of Neurobiology, Zhejiang University School of Medicine, Hangzhou, 310012 Zhejing Province China

**Keywords:** Heterotopic pancreas, Liver, Biliary tract, Hepatolithiasis, Metaplasia, Biliary epithelia cells

## Abstract

**Abstract:**

Intrahepatic heterotopic pancreas is rarely reported in the literature. Here, we report a case of a 39-year-old male with intrahepatic heterotopic pancreas associated with primary cholesterol hepatolithiasis. Computed tomography (CT) scans revealed multiple cholesterol stones in intrahepatic bile ducts of the left lobe concomitant with intrahepatic cholangiectases. These observations were confirmed by magnetic resonance cholangiopaneretography (MRCP). The patient underwent transabdominal left hepatic lobectomy. Postoperative histological examination of the resected specimen showed pancreatic tissues distributed along the wall of the bile duct and composed of acinar cells and duct elements without islets of Langerhans, therefore strongly suggesting that the heterotopic pancreas occurred in response to chronic injury due to the primary cholesterol hepatolithiasis and was derived from the biliary epithelial cells.

**Virtual Slides:**

The virtual slide(s) for this article can be found here: http://www.diagnosticpathology.diagnomx.eu/vs/1461819267158980.

## Background

Pancreatic heterotopia, which is defined as pancreatic tissues at aberrant sites and having no anatomical, neural or vascular connections with the normal pancreas [1], was first described in 1727 by Jean Schultz [2]. It is found in approximately 0.2 % surgical operations involving the upper digestive tract [3] and in 0.55 % to 13.7 % of necropsies [4]. The ectopic tissues can be located anywhere in the digestive tract and the most likely sites are the stomach (26 %–38 %), duodenum (28 %–36 %), jejunum (16 %), Meckel diverticulum, and ileum [5], while it is relatively rare in the colon, esophagus, gallbladder, bile ducts, liver, spleen, umbilicus, mesentery, mesocolon, and omentum [5]. Heterotopic pancreas is generally asymptomatic but occasionally develops into a clinical incident associated with potential complications such as inflammation, ulceration, bleeding, and obstruction [1, 6]. The location, size and pathological changes are crucial to the prediction of clinical outcomes. Here, we present a case of intrahepatic heterotopic pancreas associated with primary cholesterol hepatolithiasis in an adult male.

The article "Hepatolithiasis associated with intrahepatic heterotopic pancreas: a case report and literature review" was published in 2015. Journal: Diagn Pathol.

## Case presentation

A 39-year-old male who was diagnosed with primary cholesterol hepatolithiasis attended our out-patient department for a routine medical check-up. Further inquiry revealed a history of extracorporeal shock wave lithotripsy (ESWL) due to left ureteral calculus one year ago; no other aberrations were noted and physical examinations were normal. Liver function tests demonstrated a normal level of liver transaminases, including aspartate aminotransferase, alanine aminotransferase and γ-glutamyl transpeptidase. No clear elevation of tumor markers including α-fetoprotein (AFP), carcinoembryonic antigen (CEA), CA125 and CA-19-9 was observed. Hepatitis virus markers were all negative. Ultrasound examination showed multiple cholesterol stones in the intrahepatic bile ducts of the left lobe and hepatic steatosis. Further examinations were performed after admission of the patient to hospital. Abdominal computed tomography (CT) scans revealed several round high-density shadows within the intrahepatic biliary tract of the left lobe, which was noticeably dilated (Fig. 1a and b). A low-density mass with an estimated magnitude of 2.0 × 1.8 cm and a vague margin was also observed in the CT scan. The mass was located in the right hepatic lobe and showed signal enhancement around the wall in arterial phase, gradual enhancement toward the central area of the lesion in the portal venous and delayed phases (Fig. 1c and d). No other abnormalities were noted. Magnetic resonance cholangiopaneretography (MRCP) demonstrated multiple T2 low signal intensity foci in the left intrahepatic bile duct concomitant with cholangiectases. At the request of the patient and to rule out the possibility of cancer, a transabdominal radical excision was performed based on the clinical diagnosis of hepatolithiasis and the left hepatic lobe was successfully removed. Postoperative recovery was uneventful.

**Fig. 1:** Abdominal computed tomography scan before surgery. **a–b**: Abdominal computed tomography scan (plain and arterial phase) revealed multiple cholesterol stones in intrahepatic bile ducts of the left hepatic lobe concomitant with intrahepatic cholangiectases; **c–d**: A low-density mass (arrow) with an estimated magnitude of 2.0 × 1.8 cm and a vague margin was also observed

Gross examination showed a few yellowish-white biliary calculi within the left hepatic lobe and distinct strictures of several biliary tracts. The dilated bile ducts had a maximum circumference of 1.2 cm. Histological examination of the resected specimen showed pancreatic tissues distributed along the wall of the bile duct and composed of acinar cells and duct elements without islets of Langerhans (Fig. 2a). The acinar cells contained eosinophilic granules (Fig. 2b). The pathological diagnosis was intrahepatic cholangiectases with hepatolithiasis concomitant with pancreatic heterotopia.

The article "Hepatolithiasis associated with intrahepatic heterotopic pancreas: a case report and literature review" was published in 2015. Journal: Diagn Pathol.

**Fig. 2:** Histological examination showed pancreatic tissues distributed along the wall of the bile duct. **a**: The pancreatic tissues consisted of acinar cells and duct elements [hematoxylin and eosin (HE), ×4]; **b**: The acinar cells contained eosinophilic granules (HE, ×20)

## Discussion

The presentation of heterotopic pancreas is generally clinically silent and lacks specific preoperative diagnostic methods [7]. The possible symptoms are commonly nonspecific including abdominal pain (45.5 %), epigastric discomfort (12.0 %), nausea and vomiting (9.6 %), bleeding (8.0 %), and others signs (24.5 %) [8]. The diagnosis of the heterotopic pancreas is almost completely dependent on postoperative histological examinations, which leads to uncertainty in the clinical treatment strategy. Despite controversy, radical excision is universally considered to be the most valid treatment for the purpose of avoiding potential complications including inflammation, ulceration, bleeding, and obstruction [1, 6]. While heterotopic pancreas can be found anywhere inside the alimentary canal, the stomach, duodenum and jejunum are the most commonly reported sites [5], while other sites such as the Meckel diverticulum, ileum, are rare, and the colon, esophagus, gallbladder, bile ducts, liver, spleen, umbilicus, mesentery, mesocolon, and omentum [5] are almost completely unknown.

Confirmed cases of intrahepatic heterotopic pancreas are relatively rare and, to the best of our knowledge, only eleven incidents have been reported to date in association with cirrhosis [9], adenocarcinoma arising from intrahepatic heterotopic pancreas, hepatic and extrahepatic choledochal cysts, necropsy, Caroli’s disease, hepatic mass, insular carcinoma probably arising from intrahepatic heterotopic pancreas (1 case each), and two cases of primary cholesterol hepatolithiasis [10].

The pathogenesis of heterotopic pancreas remains to be fully clarified although three promising hypotheses had been presented to date. The first hypothesis suggests that the heterotopic pancreas arises from the separation and migration of heterotopic pancreatic tissue from the primitive pancreas during embryonic rotation [6]. The second hypothesis suggests that pancreatic metaplasia of endodermal tissues is the cause of the heterotopic pancreas [11]. Finally, it has been suggested the heterotopia is caused by abnormalities in the Notch signaling system [12, 13].

The article "Hepatolithiasis associated with intrahepatic heterotopic pancreas: a case report and literature review" was published in 2015. Journal: Diagn Pathol.

On the basis of the these three hypotheses and the currently available literature, we speculated that, due to the histological and functional features of the heterotopic pancreatic tissues, the active pancreatic enzymes secreted into the bile ducts cause recurrent inflammation, hyperplasia and dysplasia of the mucosa [14, 15]. The reconstruction of original anatomical structure and focal strictures facilitate lithogenesis which may, ultimately lead to cholelithiasis or hepatolithiasis [14, 15].

However, in the case presented here, we noticed that the heterotopic pancreatic tissues were distributed along the wall of the biliary tract and were composed of acinar cells and duct elements without islets of Langerhans. These features are distinctly different from those presenting as solitary nodules or masses. Thus, this unique histological distribution was quite difficult to interpret solely as a developmental disorder. We also noted chronic inflammation of the mucosa and mild-to-moderate epithelial dysplasia in same location in biliary tract. Previous reports indicate that intrahepatic biliary epithelial cells are able to serve as progenitors in response to certain stimuli [16]. Combined with the fact that intrahepatic bile ducts and the pancreas shared a common embryologic derivation from the caudal portion of the foregut, these findings indicate the possibility that the heterotopic tissues is derived from metaplasia of the biliary epithelium. The primary hepatolithiasis constantly irritated the biliary epithelium, eliciting recurrent local inflammation. This chronic mechanical and chemical injury induces the hyperplasia and dysplasia of the epithelium, eventually leading to transdifferentiation of the epithelial cell and pancreatic metaplasia. The exocrine pancreatic metaplasia releases secretory products, which exacerbate the inflammation and metaplasia, causing a “vicious circle” of pathological changes, finally resulting in the exacerbation of primary hepatolithiasis.

We propose that the intrahepatic heterotopic pancreas found in the case presented here occurred in response to chronic injury due to the primary hepatolithiasis. Similar instances have been described both in clinical cases and experimental reports. Wolf *et al.* [9] presented a case of liver cirrhosis, in which the heterotopic pancreatic tissues had a close relationship with proliferation of bile dutucles, therefore, strongly suggesting that the pancreatic tissues were formed by metaplasia of the biliary epithelium. Fang-Ying *et al.* [17] described 16 cases of liver explants containing pancreatic acini-like tissue, which were almost always accompanied by or intermixed with bile ductular conditions. This suggested that the pancreatic acini-like tissue was the metaplastic product of bile ductular regeneration. The experimental conversion of liver to pancreas has been widely reported [18–21]. More specifically, Masaki *et al.* [22] transfected intrahepatic biliary epithelial cells with adenoviral-pancreas duodenum homeobox 1 (Ad-Pdx-1), NeuroD or Pdx-1/VP16 *in vitro*, showing a subpopulation of these cells successfully acquired the ability to differentiate into β-cell. Although the heterotopic cells found in our study were not identical to β-cells, considering the common embryologic derivation of these cells, we suggest that it is completely feasible for intrahepatic biliary epithelial cells to be induced to differentiate into pancreatic cells.

The article "Hepatolithiasis associated with intrahepatic heterotopic pancreas: a case report and literature review" was published in 2015. Journal: Diagn Pathol.

## Conclusions

Intrahepatic heterotopic pancreas associated with primary cholesterol hepatolithiasis is rarely seen in clinical practice, not only due to the limitation of specific markers and detection methods, but also because of lack of information and vigilance. Based on the case reported here, except for the known hypotheses, our hypothesis may add to the currently proposed hypotheses and provide a new perspective for understanding the genesis of heterotopic pancreas.

### Consent

Written informed consent was obtained from the patient for publication of this Case Report and any accompanying images. A copy of the written consent is available for review by the Editor-in-Chief of this journal.

## Abbreviations

CT: Computed tomography
MRCP: Magnetic resonance cholangiopaneretography
ESWL: Extracorporeal shock wave lithotripsy
AFP: α-fetoprotein
CEA: Carcinoembryonic antigen
Ad-Pdx-1: Adenoviral-pancreas duodenum homeobox 1
